# Identification of Sports Athletes Psychological Stress Based on *K*-Means Optimized Hierarchical Clustering

**DOI:** 10.1155/2022/6555797

**Published:** 2022-08-18

**Authors:** Jun Huang

**Affiliations:** School of Competitive Sports, Shandong Sport University, Rizhao 276800, China

## Abstract

In order to solve the problem, the psychological identification of athletes in professional competition pressure is difficult. This paper first analyzes the sources of athletes' psychological pressure based on the hierarchical clustering method, and then divides the weights of the sources of psychological pressure, quantificationally scores them and constructs an identification model of athletes' psychological pressure. Then, the clustering process is optimized based on the K-Means algorithm, and its effectiveness is verified. Finally, the psychological stress of 10 players in a football club was analyzed. The results show that the model effectively and reasonably reflects the influence of pressure sources on the athletes' competitive state during the competition, which provides a basis for the decision-making of relief about athletes' stress.

## 1. Introduction

Competitive sport is a highly stressed profession that high-level athletes often lose in major competitions. With the professionalization of sports and the improvement of athletes' psychological requirements, it is an inevitable trend to relieve the pressure before competition. Therefore, it is very important to identify the stress sources of athletes in sports competitions. Psychological counseling is generally to evaluate the athletes' psychological state by consulting professionals or using some questionnaires [1, 2], where professionals divide the results given by athletes into three grades: high, medium, and low. Different grades give different psychological analysis, and generally, athletes' psychology only needs to be roughly classified according to grades [3]. To alleviate the chronic stress of athletes, team doctors and psychologists need to intervene through investigation and interviews where athletes' thoughts can be understood, and the types of stress can be identified through professional psychological analysis. In the past, the research conclusions often focused on the coping strategies of athletes in a specific event, or on a certain element or link in the coping process, so it is impossible to effectively analyze the overall psychological situation [4, 5]. When the number of athletes increases, psychologists cannot effectively make personalized judgments according to their personal situation, which is inefficient and the coping strategies and results are not ideal.

The work required for stress relief includes information collection of athletes, identification of stress sources, evaluation of sports psychological state, and formulation of strategies, among which the identification of stress sources generally includes training activity test, team doctor inquiry, real-time evaluation, and self-explanation [6]. For the work of relieving athletes' precompetition stress, source identification is the most basic and the most difficult part to implement, which is determined subjectively by the experience of team doctors, whose uncertainty is high. In the process of identifying the source of athletes' stress, because athletes' own experiences are different and their psychological feedback is different, it is particularly important to deal with the collected psychological index data reasonably. Hierarchical clustering method is a common method in the field of data mining. By grouping data samples, it can quickly summarize the common points of different cluster information and then identify the core information. In addition, it is simple, clear-thinking, and can effectively deal with big data sets, so it has been applied in many fields. However, from the perspective of identifying athletes' stress sources, the judgment chain of the hierarchical clustering method is still insufficient to deal with relevant data [7, 8].

In order to help psychological experts provide scientific suggestions, this paper carries out automatic simulation from the aspect of data mining, analyzes athletes' psychological pressure by using the clustering algorithm and effectively reflects the influence of pressure sources on the athletes' competitive state in the process of competition, which offers a basis for the formulation of decisions to athletes' stress relief.

## 2. Identification of the Athletes' Psychological Pressure Based on the Hierarchical Clustering Method

### 2.1. Clustering Algorithm

Clustering analysis is one of the main methods of data mining, which is used to divide a large number of datasets into several clusters. Typical clustering mainly includes the processes of raw data preparation, feature extraction, proximity measurement, clustering or grouping, and clustering result evaluation [9].  Figure 1 depicts the typical sequence of the first three steps, which includes a feedback route; among them, the output of grouped results will affect the extraction of data features and the calculation of its similarity:

1. Primary data preparation. It means preparing data, including processed valid data, number, quantity, type and scale of valid data, standardization, and dimension reduction of data features.
2. Feature extraction. Extracting the most effective feature subset from the original feature set to form a new dataset. Therefore, feature extraction is a method of converting the original feature subset into a more significant new feature subset to make the clustering effect more obvious.
3. Proximity measurement defines the distance function between pairs of data, which is used to measure the similarity between data;
4. Clustering or grouping. For grouping or clustering, you can use a variety of clustering algorithms, such as hard clustering (giving a clear division result) or fuzzy clustering (giving the membership degree of each data in the cluster), and hierarchical clustering algorithm.
5. Evaluation of clustering results. Evaluate whether the clustering results are valid by measuring the matching degree of clusters to data or by measuring the matching degree of clusters to benchmarks. The main evaluation methods are the object matching degree and related test evaluation.

### 2.2. Hierarchical Clustering Algorithm

Hierarchical clustering method is a common method to test abnormal data in samples which firstly standardizes multidimensional datasets and then aggregates data categories according to different levels, so that data subsets at different levels have certain similarities, while the gaps between subsets are relatively obvious [10]. According to the difference of hierarchical decomposition methods, it can be further divided into two categories: condensation and classification. Condensation clustering method takes each unit object as an independent cluster and then merges the nearest cluster in turn until the basic conditions set by the system are met or all objects are merged into one cluster. The rule of classification clustering is to treat all units of objects as a cluster and divide each cluster by iteration until the basic conditions set by the system are met or each object is divided into a cluster. Therefore, this method is also called the top-to-bottom clustering method.

### 2.3. Cluster Analysis Model

In contrast, the operation process of the aggregation clustering method is simpler, which is more suitable for the analysis of the athletes' psychological state. Therefore, this paper adopts this method. The specific clustering process is shown in Figure 2:

(1) Calculate the Euclidean distance between two clusters as
  (1) $$\begin{array}{c} d\left(i,j\right)=\sqrt{\overset{m}{\underset{i=1}{\sum }}{\left(x_{il}-x_{jl}\right)}^{2}}, \end{array}$$
where *d*(*i*, *j*) represents the distance between *x*_*i*_ and *x*_*j*_, which are composed of *m* attributes; *x*_*il*_ and *x*_*jl*_ represent the ith attribute value of *x*_*i*_ and *x*_*j*_, respectively.
(2) Construct pressure transmission.
The clustering method based on Euclidean distance is efficient, but the Euclidean distance is not transitive, that is, through *d*(*i*, *j*) > *t* and *d*(*j*, *k*) > *t*, *d*(*i*, *k*) > *t* cannot be directly deduced. In identification of athletes' stress, it is necessary to distinguish the pressure by ordinal utility theory, so that the transmission of pressure must be ensured.
Assuming that *n* object samples for {*u*_1_, *u*_2_,…, *u*_*n*_}, and each object is *m* attributes which are set as {*a*_1_, *a*_2_,…, *a*_*m*_}, and the ith object has the property of *u*_*i*_={*x*_*i*1_, *x*_*i*2_,…, *x*_in_}. Then the distance between *x*_*ik*_ and *x*_*jk*_ of the kth attribute of *u*_*i*_ and *u*_*j*_ is
  (2) $$\begin{array}{c} d_{k}\left(i,j\right)=\frac{\left|x_{ik}-x_{jk}\right|}{a_{k\max}-a_{k\min}}. \end{array}$$
Among them, *a*_*k*max_ and *a*_*k*min_, respectively, represent the maximum and minimum values of the kth attribute *a*_*k*_ of each object.
(3) Calculate the similarity of attributes.
The similarity of each attribute of object *u*_*i*_ and *u*_*j*_ is
  (3) $$\begin{array}{c} d\left(i,j\right)=\frac{\sqrt{\sum_{l=1}^{m}d_{k}^{2}\left(i,j\right)}}{m}, \end{array}$$
where, *d*(*i*, *j*) represents the distance between *x*_*i*_ and *x*_*j*_, which are composed of *m* attributes; *x*_*ii*_ and *x*_*j*_ represent the lth attribute value of *x*_*i*_ and *x*_*j*_, respectively.
  (4) $$\begin{array}{c} s\left(i,j\right)=1-d\left(i,j\right), \end{array}$$
where, *d*(*i*, *j*) represents the distance between *x*_*i*_ and *x*_*j*_.
(4) Construct similarity matrix.
The transitive closure *T* = *T*(*R*) of similarity matrix S is obtained by the quadratic method in fuzzy mathematics.
(5) Obtain a clustering result.

The corresponding clustering results can be obtained by establishing the system clustering graph based on *T* and setting a threshold value for interception.

### 2.4. Identification of Athletes' Psychological Pressure

The psychological conditions of athletes in different categories of events are selected as basic samples, and the scores of psychological pressures are taken as attributes. The above clustering analysis model is used to analyze the psychological pressures of athletes, so as to identify the clustering results of various pressures. The formula of identification is

(5) $$\begin{array}{c} Q=\frac{\left(\sum_{i=1}^{m}w_{i}e_{i}\right)}{\sum_{i=1}^{m}w_{i}}, \end{array}$$

where *m* represents the type of pressure source, *w*_*i*_ represents the score weight from sources of category *i*, which is directly related to its impact on performance. The stronger the correlation between psychological stress and the performance of the field, the higher the weight, otherwise, the lower the weight. According to “Psychological Instruction Manual for Active Athletes,” the weights are distributed and calculated in the form of index. The results are shown in Figure 3:

Among them, *n* represents the repeated times of the same kind of pressure in different athletes' psychological information.

The description of athletes under different psychological stress scores is shown in Figure 4:

## 3. Optimized Model of Athletes' Psychological Stress Based on the K-Means Algorithm

### 3.1. Optimization Process

Because the amount of data is small, and there are many features of them, if only a clustering algorithm is used, the discrimination between data will be low. In order to obtain better initial center and time complexity, the above model is improved in a hierarchical way.

Assuming that *X*={*x*_1_, *x*_2_,…, *x*_*n*_} is the data of *n* r-dimensional spaces. Firstly, the algorithm uses a contour coefficient to determine the approximate number of clusters. After hierarchical clustering is used to reach this level, the number of clusters and the initial center of iteration are locally adjusted, thus greatly saving the computation for clusters with more levels. In addition, when adjusting the initial center locally, the evaluation standard of intra-class similarity is adopted, the cluster with the lowest similarity is decomposed into two new clusters. In this way, the clusters with insufficient cohesion but mistakenly classified into one class can be adjusted locally, which makes the selection of initial center more reasonable and convenient for operation. The specific implementation steps are shown in Figure 5:

1. Data processing is carried out on the original data, and the contour coefficient is calculated. The maximum K is taken as the initial value.
2. Two adjacent clusters are combined by using the aggregation hierarchical clustering algorithm to form a new cluster.
3. The mean values of two cluster centers at the same level on the new cluster center after merging are calculated.
4. Repeat step (2) and step (3) until (*K* − *R*)(0 < =*R* < *K* − 2) cluster (if *k*=2, then *R*=0).
5. Calculate the intra-cluster similarity of all the divided clusters, respectively.
6. Select the cluster with the smallest similarity in the cluster, that is, the cluster with the largest class radius, decompose the cluster and find out the sample point *x*_*i*1_ farthest from the center *c*_*i*_ of the class, and then select the sample point *x*_*i*2_ farthest from *x*_*i*1_ in the class.
7. *x*_*i*1_, *x*_*i*2_ and other cluster centers are used as new cluster centers to make K-Means clustering again.
8. If the centroid changes, return to step (6), otherwise, the algorithm ends and the result is output.

It can be seen that from step (1) to step (4), the hierarchical clustering algorithm is used to cluster the original data; while from step (5) to step (6), K-Means clustering is started where the number of clusters is reselected according to the number of clusters roughly calculated by the previous hierarchical clustering algorithm, and the initial clustering center of the K-Means algorithm is selected according to hierarchical clustering. Finally, K-Means algorithm is used for secondary clustering from steps (7) to (8).

### 3.2. Validation of the Model

#### 3.2.1. The Validation Environment

In order to verify the effectiveness of the improved algorithm, Iris data, Breast Cancer data, and Abalone data in the UCI database are selected for verification. The size of the dataset and the number of clusters are shown in Table 1.

The experiment is tested on a PC (2.4 GHz Intel CPU, 2G memory, windows7 system). The programming language is *R* language, which is an open source language and the operating environment for statistical analysis and drawing. But it has stronger statistical analysis and data operation (especially in vector and matrix operation) functions than C language. Therefore, in this paper, the algorithm is implemented with its powerful extended language package and function of matrix calculation [11, 12].

#### 3.2.2. Validation Results

The results of clustering are compared from the aspects of operation efficiency and the aggregation degree. The comparison of CPU runtime under different models is shown in Figure 6.

It can be seen from the data that with the increase in datasets, the CPU run time increases significantly. This is because the improved algorithm uses the contour coefficient to predict the value of K in advance, and only performs small-scale optimization near the K value, which effectively reduces the time complexity of the algorithm.

In addition, in order to represent the clustering degree of the cluster, we evaluate the effectiveness of the algorithm through the accuracy rate, and the results are shown in Figure 7.

The accuracy of the improved clustering algorithm is higher than that of the traditional clustering algorithm, which shows that the efficiency and accuracy of the improved algorithm are significantly strengthened for small sample datasets.

## 4. Case Analysis

### 4.1. Index Selection

Taking the players in a football club as the research object where 10 players of different ages were randomly selected for psychological stress analysis. The participants were evaluated with the stress perception scale and the psychological stress tolerance test. The original test data were standardized as the score data of [0, 10] by using the linearization processing, then the identification model of athletes' psychological pressure in Section 4 can obtain the data of psychological stress of athletes in the club, as shown in Table 2.

There are two types of pressure sources [13]: acute pressure and chronic pressure. In specific application, the pressure sources can be further subdivided, and then the corresponding analysis is conducted by using the clustering method, so as to provide reference for the team to relief athletes' pressure.

### 4.2. Analysis of Athletes' Psychological Pressure

Taking the score data of athletes' psychological pressure under different factors into the algorithm mentioned above, the transfer closure matrix *T* of each influencing factor can be calculated as follows:

 
*T*_1_ = [1, 0.8, 0.9, 0.9, 0.8, 0.9, 0.9, 0.9, 0.9, 0.9]^*T*^
 
*T*_2_ = [0.9, 1, 0.9, 0.8, 0.8, 0.8, 0.8, 0.8, 0.8, 0.8]^*T*^
 
*T*_3_ = [0.9, 0.9, 1, 0.9, 0.8, 0.9, 0.8, 0.8, 0.8, 0.8]^*T*^
 
*T*_4_ = [0.9, 0.9, 0.9, 1, 0.9, 0.9, 0.9, 0.8, 0.8, 0.8]^*T*^
 
*T*_5_ = [0.9, 0.9, 0.9, 0.9, 1, 0.9, 0.9, 0.8, 0.8, 0.8]^*T*^
 
*T*_6_ = [0.9, 0.9, 0.9, 0.9, 0.9, 1, 0.9, 0.9, 0.8, 0.8]^*T*^.

Therefore, the system clustering diagram of this model is shown in Figure 8:

According to the transitive closure *T*, it is necessary to take 0.90 as the threshold value of the system clustering diagram. Thus, A1 and A2 are combined into a cluster, A4 and A5 are combined into a cluster, and A3 and A6 are formed into a cluster, respectively. Therefore, the psychological pressure of athletes in the club is shown in Table 3.

It can be seen from the above data that 67.87% of athletes' pressure comes from the outside, which is chronic pressure; while 32.13% of them comes from competitions, which is acute pressure. Generally speaking, athletes cannot fully concentrate in the game, and they are easy to be affected by off-site factors. To deal with a large proportion of off-site pressure, the organizers need to assist the team operators to introduce professional psychologists for counseling, so that athletes can focus on the competition.

Through the analysis of the example shows that the athletes clustering algorithm can realize effective pressure source identification, through the study of the automatic classification of athletes psychological pressure information, based on individual rating of athletes get event athletes overall pressure source, for the organizers to provide guidance for alleviating the psychological pressure of the athletes.

Athletes A2, A3, A6, and A9 have less pressure on training and life, which indicates that they have better control of tenacity, lower confidence, and enthusiasm in engagement. In addition, their overall relationship with coaches is better, but it is poor in terms of complementarity that mainly refers to the state of athletes under the guidance. The overall stress level of these athletes is relatively low which shows that they have better psychological quality, higher happiness, and social support.

## 5. Conclusion

In this paper, an analysis model of athletes' psychological pressure is constructed by the clustering algorithm, and the source of athletes' psychological pressure is identified quantitatively. The validation results show that the optimized psychological pressure analysis model can effectively reduce the time complexity of the algorithm, improve its operation efficiency and accuracy, and can better adapt to the test of psychological stress. In addition, the result of case analysis shows that the overall stress level of athletes A2, A3, A6, and A9 is relatively low, which indicates that they have better psychological quality, higher happiness, and social support. To sum up, the model realizes the automatic evaluation of athletes ‘pressure and can be used as an assistant tool for team doctors or psychologists. From a practical point of view, the pressure source identification tool constructed in this paper is practical in large-scale competitions, and the identification of athletes' pressure sources can help each team to pretest athletes' psychological pressure, and then make targeted adjustments, which is conducive to maximizing athletes' potential for competition.

## Figures and Tables

**Figure 1:** The process of the clustering algorithm.

**Figure 2:** Clustering process of athletes' psychological stress analysis.

**Figure 3:** Score weight of psychological stress sources.

**Figure 4:** Score of athletes' psychological stress.

**Figure 5:** Optimization process based on K-Means.

**Figure 6:** Comparison of CPU run time of different algorithms.

**Figure 7:** Comparison of accuracy under different algorithms.

**Figure 8:** System cluster diagram.

**Table 1:** Experimental data set.

	Size of dataset	Number of clusters
Iris	150	3
Breast cancer	300	2
Abalone data	4000	30

**Table 2:** Psychological pressure scores of athletes under different factors.

Athletes	M1 training	M2 life	Developing M3	M4 family	M5 social networking	M6 score
A1	7.44	4.56	4.48	7.98	3.45	7.89
A2	3.15	7.38	7.26	5.01	6.38	5.06
A3	4.61	3.80	3.86	8.93	3.60	8.43
A4	7.05	4.55	8.78	4.44	4.43	6.61
A5	3.19	4.94	3.15	6.27	7.07	5.65
A6	8.42	8.29	4.55	3.72	7.31	5.61
A7	8.05	3.16	8.26	8.08	4.61	5.46
A8	8.68	6.63	5.90	6.10	6.53	6.53
A9	8.77	7.84	7.34	5.88	4.92	8.81
A10	7.87	3.13	8.98	8.36	6.53	7.68

**Table 3:** Analysis of athletes' psychological pressure.

Athletes	Stress score	Relevance
A1	0.6	B
A2	1	B
A3	1	A
A4	0.7	C
A5	0.7	B
A6	1	C
A7	0.8	A
A8	0.6	A
A9	1	B
A10	0.7	C

## Data Availability

The dataset is available from the corresponding author upon request.
